# Effect of Alteplase Thrombolysis on Coagulation Function and Nerve Function of Patients with Ischemic Stroke

This article has been retracted.

**DOI:** 10.1155/2022/9440271

**Published:** 2022-05-09

**Authors:** Hong-Ying Zhao, Guo-Tao Yang, Hui-Fang Zhang, Wen-Hao Wang

**Affiliations:** ^1^Department of Geriatrics, Cangzhou Central Hospital, Cangzhou 061000, Hebei, China; ^2^Department of Neurology, Cangzhou Central Hospital, Cangzhou 061000, Hebei, China

## Abstract

**Objective:**

To investigate the effects of alteplase thrombolysis on coagulation function and nerve function of patients with ischemic stroke.

**Methods:**

76 cases with ischemic stroke receiving thrombolytic therapy in Cangzhou Central Hospital from November 2018 to November 2019 were recruited. They were assigned via the random number table method at a ratio of 1 : 1 to receive alteplase thrombolysis either within 3h after the onset (observation group) or within 3–4.5 h after the onset (control group), followed by aspirin administration after no bleeding in cranial computed tomography (CT). Outcome measures included plasma fibrinogen (FIB), activated partial prothrombin time (APTT), platelet (PLT) levels, the National Institute of Health stroke scale (NIHSS) score, and adverse events.

**Results:**

Alteplase thrombolysis within 3 h was associated with better prothrombin time (PT), APTT, FIB, and PLT levels versus thrombolysis within 3–4.5 h (*P* < 0.05). Thrombolysis within 3 h showed significantly lower NIHSS scores versus within 3–4.5 h (*P* < 0.05). The two groups showed a similar incidence of adverse events (*X*^2^ = 2.963, *P*=0.615).

**Conclusion:**

Alteplase thrombolysis showed benefits in mitigating the coagulation function and nerve function damage of patients with ischemic stroke, especially within 3 hours after the onset, with a high safety profile.

## 1. Introduction. 

Cerebrovascular diseases are the top cause of death among life-threatening diseases and are also the primary factor of disability [1]. Approximately, 70% of stroke patients in China are ischemic stroke patients, and carotid stenosis is an important cause of ischemic stroke [2, 3]. Thrombolysis is the mainstay of treatment for ischemic stroke. Ischemic stroke requires timely and effective treatment after its onset [4]. Alteplase is a tissue-type plasminogen activator that is commonly used for ischemic stroke after the exclusion of intracranial hemorrhage by imaging [5]. The results of the 1996 US NIDDS trial suggested considerable benefits of alteplase intravenous thrombolysis for acute cerebral infarction within 3 h of onset in reducing disability and improving prognosis, and the ECASS trial indicates an excellent prognosis with intravenous thrombolysis at 3.0–4.2 h after acute ischemic stroke attack. In recent years, a growing body of evidence has demonstrated promising outcomes of effective alteplase thrombolysis with the earlier use the better the prognosis [6]. However, no consensus on the timing for thrombolysis has been obtained in previous studies. Accordingly, 76 cases with ischemic stroke receiving thrombolysis in Cangzhou Central Hospital from November 2018 to November 2019 were recruited to investigate the efficacy of alteplase thrombolysis and provide a clinical reference for future treatment.

## 2. Materials and Methods

### 2.1. General Information

In this prospective study, 76 cases with ischemic stroke receiving thrombolytic therapy in Cangzhou Central Hospital from November 2018 to November 2019 were recruited. They were assigned via the random number table method at a ratio of 1 : 1 to an observation group or a control group. The clinical baseline characteristics of the observation group (21 males, 17 females, aged 60–86 (67.3 ± 4.5) years, National Institute of Health stroke scale (NIHSS) score of 4–21 (12.28 ± 4.06) points, 16 cases of hypertension, 13 cases of diabetes, and 7 cases of hyperlipidemia) were comparable with those of the control group (20 males, 18 females, aged 61–85 (67.6 ± 4.8) years, National Institute of Health stroke scale (NIHSS) score of 5–20 (12.57 ± 3.92) points, 17 cases of hypertension, 14 cases of diabetes, and 7 cases of hyperlipidemia) (*P* > 0.05). This study was reviewed by the hospital ethics committee (no. 2017-06-12), and all patients and families provided written informed consent.

### 2.2. Inclusion and Exclusion Criteria

Inclusion criteria are as follows: (1) patients met the diagnostic criteria of acute ischemic stroke, including no intracranial hemorrhage observed by CT or magnetic resonance imaging (MRI); (2) aged ≥60 years; (3) with onset time < 45 h and all patients showed no early large-area infarction; (4) with the indications for alteplase thrombolytic therapy and an NIHSS score of ≥ 4 points at the time of onset; and (5) with complete clinical data.

Exclusion criteria are as follows: (1) patients with cerebral hemorrhage, transient ischemic attack, and asymptomatic cerebral infarction; (2) with mental abnormalities, cognitive dysfunction, or severe coma; (3) with cardiogenic embolism; (4) with low-density shadows or disappearance area of brain sulci on head CT exceeding 1/3 of the blood supply area of the middle cerebral artery; and (5) with severe heart, lung, and kidney dysfunction or severe diabetes.

### 2.3. Treatment Methods

The two groups of patients were given alteplase (Boehringer Ingelheim Pharmaceutical Co., Ltd., Germany, S20110051) thrombolytic therapy at a dose of 0.9 mg/kg, and the maximum drug dose should not exceed 90 mg. Aspirin (Bayer Healthcare Co., Ltd., National Medicine Standard J20130078) was administered after no hemorrhage was found in cranial CT. The first oral dose was 0.3 g and was altered to 0.1 g/d on day 2 for long-term oral administration. Thrombolysis was performed within 3–4.5 h after the onset for patients in the control group and within 3 h after the onset for those in the observation group.

### 2.4. Outcome Measures

Before treatment and on the 10th day of treatment, fasting venous blood was collected from the patients to determine the plasma fibrinogen (FIB), activated partial prothrombin time (APTT), prothrombin time (PT), and platelet (PLT) levels of the two groups using an automatic biochemical analyzer (Myriad Mindray Automatic Biochemical Analyzer BS-350S), and the NIHSS scores were used to evaluate the neurological impairment before and after treatment. The adverse events of all patients after treatment were counted.

### 2.5. Statistical Analysis

After treatment, SPSS25.0 was used for data analyses. Measurement data were described by ($\bar{x}\pm s$). Intergroup comparison was performed using the independent sample *t*-test, and intragroup comparison was performed using the paired *t*-test. Count data were expressed in *n* (%) and subject to the *χ*2 test. The receiver operating characteristic (ROC) curve was plotted to assess the predictive value of different scoring methods for bleeding after thrombolysis. Differences were considered statistically significant at *P* < 0.05.

## 3. Results

### 3.1. Coagulation Function and Nerve Function

Before treatment, there was no marked difference in FIB, APTT, PT, and PLT between the two groups (*P* > 0.05). On the 10th day of treatment, the observation group showed significantly prolonged PT and APTT and decreased FIB and PLT versus the control group (*P* < 0.05) (Table 1).

### 3.2. NIHSS Scores

Thrombolysis within 3 h showed significantly lower NIHSS scores versus within 3–4.5 h (*P* < 0.05) (Table 2 and Figure 1).

### 3.3. Incidence of Adverse Events

The incidence of adverse events during treatment in the observation group and control group was 15.38% (6/39) and 18.42% (7/38), respectively (*χ*2 = 2.963, *P* = 0.615) (Table 3 and Figure 2).

### 3.4. Hemorrhage Risk Prediction

After retrieving the data from PubMed, it was found that spontaneous intracerebral hemorrhage (sICH) can be predicted by the multicenter stoker survey (MSS), hemorrhage after thrombolysis (HAT), (baseline blood sugar, early infarct signs, hyperdense cerebral artery sign on admission CT, age, and NIHSS on admission (SEDAN)), (glucose at presentation, race, age, sex, systolic blood pressure at presentation, and the severity of stroke at presentation (GRASPS)), and safe implementation of thrombolysis in stroke-monitoring study (SITS) scoring systems. Their risk of bleeding after thrombolysis was compared using ROC curves. The results showed that the area under the five scoring systems exceeded 0.5, with HAT the largest. It has certain accuracy in predicting the risk of bleeding after thrombolysis.

## 4. Discussion

Ischemic stroke is a brain tissue necrosis disease caused by stenosis or occlusion of the cerebral artery. It includes transient ischemic attack (TIA), reversible ischemic neurologic deficit (RIND), and sickness impact profile (SIP). Clinical studies have shown [6–8] that ischemic stroke has high mortality and disability after treatment, which seriously compromises the prognosis of patients. After the onset of the disease, thrombolytic therapy can dredge the blocked blood vessels, which has become the treatment of choice [9–11]. Ischemic stroke can cause compression and interruption of nerve conduction pathways, resulting in clinical manifestations such as hemiplegia, aphasia, and other neurological impairments. Moreover, brain tissue hypoxia and ischemia will disrupt the blood-brain barrier and release more free radicals and inflammatory factors, resulting in a cascade of stress reactions, electrolyte, and acid-base imbalance, abnormal blood glucose metabolism, and secretion of regulatory factors, thereby compromising the body's blood rheological index. Currently, clinical treatment for stroke centers on anticoagulation or antiplatelet aggregation, plaque stabilization, blood pressure control, dehydration to lower intracranial pressure, and nutritional brain cells. However, these approaches present a poor long-term prognosis with high mortality [11]. The outcome of thrombolytic therapy is relatively poor when it is performed later than 4.5 h after the onset [12, 13].

Alteplase [14] is a synthetic tissue-type plasminogen activator (t-PA) and is produced through genetic recombination technology. It has the same properties as natural t-PA and can activate plasminogen binding to fibrin, which is converted into plasmin [15]. It is mainly used for the ablation of local fibrin clots in patients with myocardial infarction within 6 hours after onset. The main adverse reactions include coagulopathy, bleeding, hematocrit, and hemoglobin reduction. In the event of severe bleeding, fresh freeze-dried plasma or fresh whole blood is required, and synthetic antifibrinolytic agents are also applied when necessary. The blood concentration of alteplase varies in different individuals which is attributed to the different liver blood flow and PAI-1. Abnormal coagulation function in patients with ischemic stroke contributes to thrombus formation by the abnormal release of coagulation substances. Alteplase is a thrombolytic agent that targets fibrin specifically and activates fibrinogen to fibrinolytic enzymes, thus disrupting the fibrin meshwork in the thrombus and exerting a good thrombolytic effect [16, 17].

The results of the present study showed that alteplase thrombolysis within 3 h was associated with better PT, APTT, FIB, and PLT levels and lower NIHSS scores versus thrombolysis within 3–4.5 h, and the two groups showed a similar incidence of adverse events. All these confirm that the use of alteplase thrombolysis in elderly patients with ischemic stroke can improve coagulation function and reduce neurological damage, with a promising safety profile especially performed within 3 hours after the onset. The reason may be that the thrombolytic therapy implemented in the initial stage of cerebral ischemia can promote blood perfusion of brain tissue and reduce nerve damage caused by the insufficient blood supply to brain tissue. In addition, aspirin was used for treatment after thrombolysis. Its long-term use can prevent the formation of thromboxane A2 by inhibiting the prostaglandin epoxidase of platelets, thereby inhibiting platelet aggregation, preventing the formation of thrombus, and improving the coagulation function.

## 5. Conclusion

Alteplase thrombolysis showed benefits in mitigating the coagulation function and nerve function damage of patients with ischemic stroke, especially within 3 hours after the onset, with a high safety profile. The limitation of this study is that this study is a single-center study with a small sample size, which may result in bias. Future randomized, multicenter, large-sample size studies are required to provide better treatment alternatives for patients.

## Figures and Tables

**Figure 1:** Comparison of NIHSS scores between the two groups at different times.

**Figure 2:** ROC curves of different scoring methods for predicting bleeding after thrombolysis.

**Table 1:** Comparison of the coagulation function of the two groups of patients before and after treatment ($\bar{x}\pm s$).

Groups	Time	FIB (g/L)	APTT (s)	PT (s)	PLT (×10^9^/L)
Treatment group (*n* = 38)	Before treatment	3.42 ± 0.68	24.32 ± 0.35	9.63 ± 0.78	321.57 ± 22.46
	10 d after thrombolysis	2.35 ± 0.45^*∗*^^#^	28.76 ± 2.35^*∗*^^#^	11.59 ± 0.93^*∗*^^#^	167.59 ± 11.42^*∗*^^#^

Control group (*n* = 38)	Before treatment	3.41 ± 0.65	24.34 ± 0.32	9.65 ± 0.73	322.16 ± 23.54
	10 d after thrombolysis	3.15 ± 0.52^*∗*^	25.74 ± 2.18^*∗*^	10.58 ± 0.84^*∗*^	254.79 ± 15.46^*∗*^

Compared with before treatment, ^*∗*^*P* < 0.05; compared with the control group, ^#^*P* < 0.05.

**Table 2:** Comparison of NIHSS scores between the two groups before and after treatment.

Groups	Before treatment	24 h after thrombolysis	10 d after thrombolysis
Treatment group (*n* = 38)	12.28 ± 4.06	8.47 ± 1.03	6.27 ± 1.14
Control group (*n* = 38)	12.57 ± 3.92	11.03 ± 1.25	9.85 ± 1.56
t	8.293	3.684	2.831
*P* value	>0.05	<0.05	<0.05

**Table 3:** Comparison of the incidence of adverse reactions during treatment between the two groups of patients (*n* (%)).

Groups	*n*	Nausea and vomiting	Dizziness and headaches,	Gastrointestinal bleeding	Ecchymosis	Total incidence
Treatment group	38	2 (5.26)	1 (2.63)	1 (2.63)	2 (5.26)	15.38
Control group	38	1 (2.63)	1 (2.63)	3 (7.90)	2 (5.26)	18.42
*χ* ^2^						2.963
*P* value						>0.05

## Data Availability

The datasets used during the present study are available from the corresponding author upon reasonable request.
